The article "EZH2 Regulates ANXA6 Expression via H3K27me3 and Is Involved in Angiotensin II-Induced Vascular Smooth Muscle Cell Senescence" was retracted in 2023. Reasons: signs of a paper mill; compromised peer review; unreliable results or conclusions.

# EZH2 Regulates ANXA6 Expression via H3K27me3 and Is Involved in Angiotensin II-Induced Vascular Smooth Muscle Cell Senescence

**DOI:** 10.1155/2022/4838760

**Published:** 2022-09-14

**Authors:** Yuejin Li, Shikui Guo, Yingpeng Zhao, Rougang Li, Yu Li, Changtao Qiu, Le Xiao, Kunmei Gong

**Affiliations:** ^1^Department of General Surgery, The First People's Hospital of Yunnan Province (The Affiliated Hospital of Kunming University of Science and Technology), Kunming, Yunnan 650032, China; ^2^Department of Hepatic-Biliary-Pancreatic Surgery, The First Hospital of Kunming (The Calmette Hospital), Kunming, Yunnan 650224, China

## Abstract

**Objectives:**

Abdominal aortic aneurysm (AAA) has a high risk of rupture of the aorta and is one of the leading causes of death in older adults. This study is aimed at confirming the influence and mechanism of the abnormally expressed ANXA6 gene in AAA.

**Methods:**

Clinical samples were collected for proteome sequencing to screen for differentially expressed proteins. An Ang II-induced vascular smooth muscle cell (VSMC) aging model as well as an AAA animal model was used. Using RT-qPCR to detect the mRNA levels of EZH2, ANXA6, IK-6, and IL-8 in cells and tissues were assessed. Western blotting and immunohistochemistry staining were used apply for the expression of associated proteins in cells and tissues. SA-*β*-gal staining, flow cytometry, and DHE staining were used to detect senescent cells and the level of ROS. The cell cycle was assessed by flow cytometry. Arterial pathology was observed by HE staining. The aging of VSMCs in arterial tissue was assessed by coimmunofluorescence for *α*-SMA and p53.

**Results:**

There were 24 differentially expressed proteins in the AAA clinical samples, including 10 upregulated protein and 14 downregulated protein, and the differential expression of ANXA6 was associated with vascular disease. Our study found that ANXA6 was highly expressed and EZH2 was lowly expressed in an Ang II-induced VSMC aging model. Knockdown of ANXA6 or overexpression of EZH2 inhibited Ang II-induced ROS, inhibited cell senescence, decreased Ang II evoked G1 arrest, and increased cells in G2 phase, while overexpression of ANXA6 played the opposite role. Overexpression of EZH2 inhibited ANXA6 expression by increasing H3K27me3 modification at the ANXA6 promoter. Simultaneous overexpression of EZH2 and the protective effect of EZH2 on cell senescence were partially reversed by ANXA6. Similarly, ANXA6 was highly expressed and EZH2 was lowly expressed in an Ang II-induced AAA animal model. Knockdown of ANXA6 and overexpression of EZH2 alleviated Ang II-induced VSMC senescence and inhibited AAA progression, while simultaneous overexpression of EZH2 and ANXA6 partially reversed the protective effect of EZH2 on AAA.

The article "EZH2 Regulates ANXA6 Expression via H3K27me3 and Is Involved in Angiotensin II-Induced Vascular Smooth Muscle Cell Senescence" was retracted in 2023. Reasons: signs of a paper mill; compromised peer review; unreliable results or conclusions.

**Conclusion:**

EZH2 regulates the ANXA6 promoter H3K27me3 modification, inhibits ANXA6 expression, alleviates Ang II-induced VSMC senescence, and inhibits AAA progression.

## 1. Introduction

AAA is a degenerative vascular complication distinguished by local dilation of the abdominal aorta to 50% of its normal diameter, which increases the risk of rupture and triggers the high morbidity and mortality worldwide [1, 2]. The prevalence of AAA is approximately 4-8% in men over 60 years old and approximately 0.5-1.5% in women [3]. In addition, other risk factors for AAA are male sex phenotype, being a member of a white race, positive family history, smoking, and atherosclerosis [4]. Pathological hallmarks of AAA are medial vascular smooth muscle cell (VSMC) depletion, reactive oxygen species (ROS) dysregulation, extracellular matrix (ECM) degradation, and inflammatory cell infiltration [2, 5]. It has been well documented that the senescence of VSMCs takes a lead in the constitution and advancement of AAA. Aging VSMCs release a category of proinflammatory cytokines and matrix-degrading molecules which benefit AAA formation [1]. Increased ROS and subsequent oxidative stress are major factors in cellular senescence, while inflammatory cytokines emitted by aging cells further trigger inflammation in encompassing tissues [6, 7].

In this study, we performed proteomic sequencing of whole aortic tissue samples from AAA patients in the anterior segment of the maximum diameter point of the intrarenal aorta and in adjacent normal tissue and found that the host protein annexin A6 (ANXA6) was highly expressed in AAA tissue. Between the membrane microdomains and the cytoskeleton, ANXA6 acts as a scaffold to function [8]. ANXA6 has been shown to be involved in sporadic cerebral cavernous malformations and mulberry poplar clusters in zebrafish [9]. At the same time, ANXA6 also promotes VSMC mineralization, thereby promoting vascular calcification [10]. Of note, vascular calcification has been recognized as a hallmark of AAA dilation [11]. Therefore, we speculate that the elevated ANXA6 in AAA tissues is related to the development of AAA.

It has been reported that ANXA6 expression is affected by H3 lysine 27 trimethylation (H3K27me3) [12]. EZH2 is an H3K27 dimethyl-and trimethyl-histone methyltransferase that mediates silencing at specific genomic loci [13–15]. In addition, EZH2 has been reported to be downregulated in AAA tissues [16]. Overexpression inhibits AAA formation and inhibits VSMC apoptosis [11]. Therefore, we conducted this study to inspect whether EZH2 affects angiotensin II- (Ang II-) induced VSMC senescence by controlling the expression of ANXA6 through H3K27me3.

The article "EZH2 Regulates ANXA6 Expression via H3K27me3 and Is Involved in Angiotensin II-Induced Vascular Smooth Muscle Cell Senescence" was retracted in 2023. Reasons: signs of a paper mill; compromised peer review; unreliable results or conclusions.

## 2. Materials and Methods

### 2.1. Patients and Tissue Samples

In this study, the samples were collected from The First People's Hospital of Yunnan Province, and the diagnostic criteria for AAA was defined as a vessel diameter greater than 1.5 times the normal vessel diameter, as determined by a vascular surgeon based on CT scans. According to the Declaration of Helsinki, the experiment was approved by the Ethics Committee of the First People's Hospital of Yunnan Province. Each patient was giving informed consent. Before resection of the AAA, ECG was performed to rule out arrhythmia, myocardial infarction, and myocardial ischemia (Figure S1). Human AAA specimens and adjacent normal tissue specimens obtained by surgery were used. The obtained samples were fixed in formalin and sent to Jingjie Biological Company (Hangzhou, China) for proteome sequencing.

### 2.2. Culture and Transfection of VSMCs

The VSMC cells were bought from the ATCC cell bank and seeded on the 10% fetal bovine serum with 1% penicillin/streptomycin and placed at 37 °C degrees and cultured under the condition of 5% CO_2_. Stimulation of VSMCs with 20 nM Ang II in complete medium for 48 h induced VSMC senescence. As the ROS scavenger, 0.6 mM N-acetyl-L-cysteine (NAC, Biyuntian, China) was added for 24 h to inhibit ROS generation. Cells treated with 10 *μ*M EZH2 inhibitor GSK126 (GIpBio, USA) were treated for 72 h to examine the effect of EZH2 on ANXA6 expression. si-ANXA6 and OE-EZH2, using GenePharma, to synthesize or construct the negative control and transfected utilizing the Lipofectamine 2000 reagent were used.

### 2.3. Western Blot

In this study, the proteins were extracted and using BCA assay (Sangon Biotech, Shanghai) to determine the total protein content. Electrophoresis experiment of total protein was carried out with 10% SDS-PAGE, and through constant current flow at 200 mA, the total protein were transferred to PVDF membrane. Subsequently, PVDF membranes were cultured with p16, p53, p21, and *β*-actin antibodies for 12 h at 4°C. Using TBS buffer, wash the PVDF membranes and incubate with secondary antibodies at room temperature for 1 h. All antibodies were purchased from abcam(UK). After washing the membrane three times, chemiluminescent reagents were added, and the bands were analyzed for grayscale values using ImageJ software. Each experiment was repeated 3 times independently.

### 2.4. RT-qPCR

In this study, we use Total RNA Extractor (Sangon Biotech) to extract the total RNA from all samples. Using cDNA synthesis kit (Vazyme, Nanjing, China), reverse transcribe 2 *μ*g mRNA into cDNA and dilute it 10 times. 1 *μ*L of the prepared cDNA was used for qPCR. Primers for IL-6, IL-8, and *β*-actin were based on designs outlined in previous studies [17]. All primers in this study were designed with Premier 5.0. The confidence of the PCR results was assessed by the dissociation curve and cycle threshold (CT) values. The results were calculated by 2^-*ΔΔ*Ct^ method after repeating over 3 times at least.

The article "EZH2 Regulates ANXA6 Expression via H3K27me3 and Is Involved in Angiotensin II-Induced Vascular Smooth Muscle Cell Senescence" was retracted in 2023. Reasons: signs of a paper mill; compromised peer review; unreliable results or conclusions.

### 2.5. ROS Levels Were Detected by Flow Cytometry

In this study, samples were lysed in 0.01 mol/L PBS and centrifuged at 500 × g at low temperature (4°C). Then, mixed with the 190 *μ*L supernatant and 10 *μ*L dichlorodihydrofluorescein diacetate (DCFH-DA; 1 M) and microtiter wells for 30 minutes at room temperature. Ultimately, the ROS levels were displayed by the ROS Assay Kit (Beyotime, Shanghai, China) as fluorescence/mg protein. Similarly, the mixture of astrocyte and 10 micron DCFH-DA incubated in 96-well plate at 25°C for 30 minutes was measured by fluorometer.

### 2.6. Senescence-Associated *β*-Galactosidase (SA-*β*-Gal) Staining

According to the instructions of the SA-*β*-gal kit (Abcam, UK) to measure senescence by SA-*β*-gal staining. Briefly, freshly isolated aortas were put with 4% paraformaldehyde for 12 h at 4°C washed and cultured for 24 hours at 37°C with staining solution. The blue SA-*β*-gal-positive cells were considered to be senescent cells and were observed using light microscopy, representing, and SA-*β*-gal-positive regions were measured by ImageJ.

### 2.7. DHE Staining

DHE staining was performed according to the literature [1]. In short, tissues of each group were collected, and ROS production in aortic slices of each group was measured using DHE (Abcam, UK), an oxidative fluorescent dye. At 37°C, the sections and cells were incubated with DHE solution for 0.5 h. Finally, ImageJ Pro software was used to measure the fluorescence intensity.

### 2.8. Cell Cycle Assessment

At room temperature, using 70% precooled ethanol fixed the cells for 12 h at 4°C in each group. Then, PI (5 mg/mL) and RNase A (100 *μ*g/mL) were used to stain for 30 minutes and analyzed by flow cytometry.

### 2.9. Laboratory Animals and Handling

15 male SD rats (age 8-10 weeks, 230-270 g/per) were bought from Hunan Slack Jingda Laboratory Animal Co., Ltd., and reared with the controlled conditions of 50% humidity, 24-26°C, and a 12 h circadian cycle. Food and water were freely available. The AAA model was established according to reference [2]: the rats were anesthetized by inhaling isoflurane (induction dose: 3-5%, maintenance dose: 1-2%), and angiotensin II (Ang II; Sigma–Aldrich, USA) or saline (sham group) was implanted into the backs of the rats (releasing a constant concentration of 1000 ng/kg/min) for 28 days. Rats died by excess CO_2_ on Day 28, and aortas of the rats were harvested for further biochemical analysis. The aorta was cleared of the adjacent connective tissue and fat and photographed on a ruler. The incidence of AAA was determined by a 50% or greater dilation of the prerenal aortic outer diameter compared to the mean maximum abdominal aortic diameter of a group of normal rats. We injected si-ANXA6 and OE-EZH2 (both 10 mg/kg) into the tail vein of Ang II-infused rats. Four injections were performed on Days 0, 7, 14, and 21 after implantation of the minipump. All animal experiments were approved by the Laboratory Animal Ethics Committee of Kunming University of Science and Technology and obtained the approval form.

The article "EZH2 Regulates ANXA6 Expression via H3K27me3 and Is Involved in Angiotensin II-Induced Vascular Smooth Muscle Cell Senescence" was retracted in 2023. Reasons: signs of a paper mill; compromised peer review; unreliable results or conclusions.

### 2.10. Immunohistochemical Staining

Immunohistochemical staining was performed according to the literature [18]. In short, 5 *μ*m sections rat abdominal aorta tissue was cut and dewaxed with xylene and rehydrated with distilled water. Then, 1% bovine serum albumin was used to block the sections for 30 min at 25°C, and the primary antibodies against ANXA6 and EZH2 were used to incubate for 12 h at 4°C. It was washed with PBS for 3 times, then the secondary antibody was used to incubate it for 4 h, and it was stained with diaminobenzidine (DAB) (Sigma–Aldrich, USA) after washing. Finally, sections were counterstained with hematoxylin to visualize nuclei. ImageJ was used to analyze the positive regions.

### 2.11. Coimmunofluorescence Staining

Coimmunofluorescence staining was used in this study according to the literature [18]. In short, 0.3% Triton X-100 in PBS was used to permeabilize the 5 *μ*m paraffin sections for 5 minutes and u 10% bovine serum albumin was used to block paraffin sections for 12 h with a p53 or ANXA6 rabbit monoclonal antibody (all 1 : 100, Abcam, UK) and then on the next day with the anti-rabbit secondary antibody (1 : 500, Abcam, UK). The sections were then cross-labeled with a secondary *α*-SMA rabbit monoclonal antibody (1 : 100, Abcam, UK) overnight and the next day with the anti-rabbit secondary antibody (Alexa Fluor 594) (1 : 500, Abcam, UK). Expect that, the tissue sections were stained with DAPI and examined by Olympus FV1000 laser confocal microscope (Olympus, Japan). Aortic fluorescence in each group was quantified using ImageJ software.

### 2.12. HE Staining

HE staining was performed according to the literature [1]. The rat femurs were fixed for 2 days, and 10% EDTA was used to decalcify with solution. The femur was taken about 1 cm in length and dehydrated with graded ethanol (70%, 80%, 90%, 95%, 100% ×3, soaking in each solution for 60-70 min). Xylene transparent (2 lanes, total 60 min), immersion wax (3 lanes, total 70 min). Routine paraffin-embedded sections. After dewaxing with xylene, it was soaked in hematoxylin staining solution for 3 min, rinsed with tap water for 10 minutes, differentiated with 1% hydrochloric acid and ethanol for several seconds, rinsed again with running water for 10 minutes until the blue color is restored, stained with eosin staining solution for 3 minutes, and rinsed for 10 minutes. Xylene was transparent, neutral resin mounts, observed under microscope and photographed.

The article "EZH2 Regulates ANXA6 Expression via H3K27me3 and Is Involved in Angiotensin II-Induced Vascular Smooth Muscle Cell Senescence" was retracted in 2023. Reasons: signs of a paper mill; compromised peer review; unreliable results or conclusions.

### 2.13. Statistical Analysis

Data are given in mean ± SD. In statistical comparison, Student's *t*-test was used when there were only two groups of differences. Moreover, one-way ANOVA was served for multiple groups depends on the usage of Student's *t*-test.

## 3. Results

### 3.1. Increased Expression of ANXA6 in AAA Tissues

Proteome analysis of infrarenal abdominal aortic tissue and adjacent normal tissue from patients undergoing elective open AAA repair revealed 24 differentially expressed proteins, 10 of which were upregulated and 14 of which were downregulated (Figures 1(a) and 1(b)). The literature has showed that the differential expression of ANXA6 is associated with vascular disease [9–11]. Therefore, we chose the highly expressed ANXA6 for our study. In the cell experiment, RT–qPCR and Western blotting were used to assess the level of ANXA6 mRNA and ANXA6 protein after treating VSMCs with Ang II and found that Ang II upregulated the level of ANXA6 mRNA and protein (Figures 1(c) and 1(d)). In addition, we used Ang II to induce the rat AAA model, and immunohistochemistry staining and Western blotting were used to assess the level of ANXA6 in AAA tissues. The level of ANXA6 was upregulated in AAA tissues (Figures 1(e) and 1(f)). In addition, we also found that ANXA6 was also expressed in vascular smooth muscle cells (Figure 1(e)). We subsequently investigated the effect of ANXA6 on VSMCs.

### 3.2. Knockdown of ANXA6 Inhibits Ang II-Induced VSMC Senescence

Because VSMC senescence is associated to the advancement of AAA, we examined the effect of ANXA6 on VSMCs senescence by ANXA6 knockdown or overexpression. After transfected with si-ANXA6, ANXA6 was significantly reduced but increased after transfected with OE-ANXA6 (Figure S2 A-B). The level of p16, p53, and p21, markers of aortic senescence, was significantly upregulated in the Ang II group. By contrast, the level of p16, p53, and p21 was significantly downregulated after ANXA6 knockdown (Figure 2(a)). In the Ang II group, the mRNA level of IL-6 and IL-8, markers of the senescence-associated secretory phenotype, was obviously upregulated. By contrast with the Ang II group, the mRNA level of IL-6 and IL-8 was obviously downregulated after ANXA6 knockdown (Figure 2(b)). Because cycle arrest is a major feature of aging, the distribution of the cell cycle phases was analyzed by flow cytometry [19]. The Ang II group demonstrated G1 arrest, and when ANXA6 was knocked down, there was decreased G1 arrest, increased G2 cells, and opposite effect in ANXA6 overexpression cells (Figure 2(c)). ANXA6 knockdown inhibits Ang II-induced VSMCs aging.

The article "EZH2 Regulates ANXA6 Expression via H3K27me3 and Is Involved in Angiotensin II-Induced Vascular Smooth Muscle Cell Senescence" was retracted in 2023. Reasons: signs of a paper mill; compromised peer review; unreliable results or conclusions.

### 3.3. Knockdown of ANXA6 Inhibits VSMC Senescence by Inhibiting Ang II-Induced ROS

It is known that ROS are the mechanism of Ang II-induced VSMC senescence [1, 20, 21], and ROS induces cell cycle arrest [22]. Therefore, we confirmed the influence of ANXA6 on Ang II-induced ROS. The flow cytometry results showed that ROS levels were significantly increased after Ang II stimulation, and ROS levels were reduced by ANXA6 knockdown or treatment with NAC, a reactive oxygen scavenger. Overexpression of ANXA6 promoted the increase of ROS induced by Ang II, and NAC partially reversed the promotion of ROS by overexpression of ANXA6 (Figure 3(a)). The Western blot results showed that the Ang II-induced upregulation of p16, p53, and p21 was mitigated by ANXA6 knockdown or by the reactive oxygen species scavenger NAC. Overexpression of ANXA6 promoted Ang II-induced upregulation of p16, p53, and p21, while NAC partially restored the role of ANXA6 overexpression(Figure 3(b)). The RT-qPCR results showed that IL-6 mRNA and IL-8 mRNA expressions were significantly upregulated in the Ang II group and that IL-6 mRNA and IL-8 mRNA were significantly downregulated after ANXA6 knockdown or treatment with the reactive oxygen scavenger NAC. Overexpression of ANXA6 promoted Ang II-induced upregulation of IL-6 mRNA and IL-8 mRNA, and NAC alleviates the increase in IL-6 mRNA and IL-8 mRNA induced by overexpression of AnxA6 (Figure 3(c)). The flow cytometry demonstrated that the G1 arrest induced by Ang II was alleviated by ANXA6 knockdown or handling with NAC, a reactive oxygen species scavenger. ANXA6 overexpression promoted Ang II-induced G1 block, and NAC alleviates this cycle arrest induced by overexpression of ANXA6 (Figure 3(d)). These results indicate that ANXA6 knockdown inhibits VSMC senescence by inhibiting Ang II-induced ROS production.

### 3.4. Knockdown of ANXA6 Inhibits VSMC Senescence by Inhibiting Ang II-Induced ROS in AAA Rats

Next, we used animal experiments to verify the effect and mechanism of ANXA6 on AAA in vivo. The effect of ANXA6 on AAA was examined after tail vein injection of ANXA6. Representative images of each group of aneurysms are shown in Figure 4(a). The quantitative analysis of the maximum diameter of the aorta showed that the outer diameter of the aorta injected with Ang II was significantly increased. Compared with the Ang II group, the aortic outer diameter was decreased after ANXA6 knockdown (Figure 4(b)). Compared with NC group, ANXA6, p16, p53 and p21 expressions were up-regulated in Ang II group, but ANXA6 knockdown reversed the above phenomenon (Figure 4(c)). In the Ang II group, the mRNA level of of IL-6 and IL-8 were increased and lower in the ANXA6 knockdown group (Figure 4(d)). The level of ANXA6 was assessed by immunohistochemistry staining. In the Ang II group, ANXA6 expression was increased but decreased in the Ang II+si-ANXA6 group (Figure 4(e)). Further, in order to specifically detect ANXA6 expression in VSMCs, we used coimmunofluorescence staining to detect *α*-SMA and ANXA6 double-positive areas. It was indicated that, in the Ang II group, the double-positive area was higher but have the opposite result in the si-ANXA6 group (Figure 4(f)). In the Ang II group, the number of positive cells was higher but was lower in Ang II+si-ANXA6 group by SA-*β*-gal staining (Figure 4(g)). In order to further verify whether VSMCs in AAA tissue has senescence, we performed VSMC markers *α*-SMA and p53 double staining. In the Ang II group, the *α*-SMA (green) and p53(red) double staining showed that the positive area of double staining was higher and that the positive area of double staining in the Ang II+si-ANXA6 group was lower (Figure 4(h)). In the Ang II group, the DHE staining proved that the positive area was higher and the positive area of the Ang II+si-ANXA6 group was lower (Figure 4(i)). The HE staining indicated that the middle elastic lamina was flattened, fragmented, and degenerated and that the aortic wall structure was fragmented in the Ang II group compared with the NC group (Figure 4(j)). Compared with Ang II, ANXA6 knockdown significantly reduced elastin degradation in the arterial media, thereby preserving the intact aortic wall structure (Figure 4(j)). In conclusion, ANXA6 knockdown inhibits VSMC senescence in vivo by inhibiting Ang II-induced ROS production.

The article "EZH2 Regulates ANXA6 Expression via H3K27me3 and Is Involved in Angiotensin II-Induced Vascular Smooth Muscle Cell Senescence" was retracted in 2023. Reasons: signs of a paper mill; compromised peer review; unreliable results or conclusions.

### 3.5. EZH2 Downregulates ANXA6 Expression via H3K27me3

Since previous studies have shown that ANXA6 expression is affected by H3K27me3 and that EZH2 is an H3K27 transferase, we next examined whether EZH2 regulates ANXA6 expression in AAA by affecting H3K27me3. The level of EZH2 and H3K27me3 at the ANXA6 promoter was assessed by ChIP-qPCR. The enrichment of EZH2 and H3K27 in the ANXA6 promoter region can be increased by overexpressing of EZH2 and that GSK126 (a selective inhibitor of EZH2 methyltransferase activity) downregulated the enhancement of H3K27 in the ANXA6 but had no significant effect on the enrichment of EZH2 at the ANXA6 promoter (Figures 5(a) and 5(b)). Expect that, GSK126 had no significant effect on EZH2 (Figure S3). Overexpression of EZH2 increased H3K27me3 expression and downregulated ANXA6, while the EZH2 inhibitor GSK126 downregulated H3K27 expression and increased ANXA6 expression (Figure 5(c)). RT-qPCR results showed that overexpression of EZH2 downregulated the ANXA6 mRNA expression and GSK126 increased ANXA6 mRNA expression (Figure 5(d)). These results propose that EZH2 downregulates the expression of ANXA6 through H3K27me3. The transfection efficiency of OE-EZH2 is shown in Figure S2C.

### 3.6. Overexpression of EZH2 Inhibits Ang II-Induced ROS and VSMC Senescence by Downregulating ANXA6 Expression

Next, we verified whether EZH2 inhibits Ang II-induced ROS production by downregulating ANXA6 expression via H3K27me3 to inhibit VSMC senescence. The results of the flow cytometry (Figures 6(a) and 6(d)), RT-qPCR (Figure 6(b)) and Western blotting (Figure 6(c)) assessed and implied that overexpression of EZH2 could hinder the increase in ROS and the senescence of VSMCs induced by Ang II. Simultaneous overexpression of EZH2 and ANXA6 partially reversed the effect of EZH2 overexpression. They proved that EZH2 overexpression inhibits Ang II-induced ROS production by downregulating ANXA6 expression to inhibit VSMC senescence.

### 3.7. EZH2 Suppresses VSMC Senescence in AAA Rats by Inhibiting ANXA6 Expression

Furthermore, we verified in rats that EZH2 regulates VSMC senescence by regulating ANXA6. A representative image of each group of aneurysms is shown in Figure 7(a). Aortic maximum diameter results (Figure 7(b)), HE staining (Figure 7(c)), SA-*β*-gal staining (Figure 7(d)), *α*-SMA and p53 double staining (Figure 7(e)), DHE staining (Figure 7(f)), immunohistochemistry staining (Figures 7(g) and 7(h)), Western blotting (Figure 7(i)), and RT-qPCR (Figure 7(j)) presented that overexpression of EZH2 can inhibit the increase of reactive oxygen species in the aorta and the aging of vascular smooth muscle cells in rats with abdominal aortic aneurysm induced by Ang II, thus weakening the progress of abdominal aortic aneurysm induced by Ang II. The protective effect of EZH2 on AAA could be partially reversed by overexpression of ANXA6. Therefore, EZH2 can inhibit VSMC senescence in AAA rats by inhibiting ANXA6 expression.

## 4. Discussion

Cellular aging is a condition triggered by a category of stress factors. Cellular senescence is characterized by loss of proliferation ability, stagnant cell cycle, apoptosis opposition, and anomalous level of secretory phenotype (SASP) factors (IL-6, IL-8, IFN-*γ*, etc.) of senescence-associated [23–26]. Senescent cells have now been detected in a group of age-related diseases [24]. It is well documented that senescence of VSMCs is engaged in the process of cardiovascular disease. Senescent cells impair essential cellular functions by modifying morphology and gene expression patterns. These alterations provoke maladjusted vascular phenotypes that enhance inflammation, thrombosis, and atherosclerosis and impair vasodilation, angiogenesis, and revascularization which contribute to the advancement of cardiovascular disease [19, 27, 28]. Several studies have found that VSMCs show cell senescence in human and rat AAA tissues and that inhibiting the senescence of VSMCs can inhibit the AAA process. [1, 5, 18] We also confirmed this by constructing an AAA rat model.

The article "EZH2 Regulates ANXA6 Expression via H3K27me3 and Is Involved in Angiotensin II-Induced Vascular Smooth Muscle Cell Senescence" was retracted in 2023. Reasons: signs of a paper mill; compromised peer review; unreliable results or conclusions.

ANXA6 appertains to a highly maintained family of annexins that are present in the plasma membrane, endosomes, and secretory vesicles for organizing membrane domains, cytoskeletal rearrangements, and the formation of signaling complexes [29–31]. Similar to other annexins, ANXA6 binds to negatively charged phospholipids, cholesterol, and nucleotides, as well as a large number of proteins in a Ca^2+^-dependent manner to activate cell membranes in a dynamic, reversible, and regulated manner [32, 33]. ANXA6 has been widely studied in cancer, but based on the type and degree of malignancy of the tumor, ANXA6 can have tumor-inhibitory activity or tumor-promoting activity [34]. We performed proteome sequencing by collecting samples from the anterior section of the maximum diameter of the intrarenal aorta in patients with AAA then found that ANXA6 was highly expressed in AAA tissue. In addition, we also found that VSMCs could be induced by Ang II, and the expression of ANXA6 was highly expressed in rat AAA tissues. Knockout of ANXA6 can inhibit the increase of ROS induced by Ang II and the aging of VSMCs, thus alleviating the pathogenesis of AAA.

Epigenetics is usually described as changing gene expression without changing DNA sequence, which is a genetic and acquirable genome modification. In some cases, epigenetic modifications exist stably and can be passed on to offspring, but many modifications occur relatively dynamically and can make corresponding biological responses to environmental cues [35, 36]. Histones can undergo dynamic chemical modifications, including methylation, acetylation, phosphorylation, and ubiquitination, as their N-termini are exposed on the surface of nucleosomes [13]. Histone methylation is a posttranslational process in which methyl groups are linked to H3 and H4 proteins by the enzyme histone methyltransferase (HMT), thereby altering the interaction of histones with DNA and nuclear proteins. Depending on the methylation site and its effect on chromatin structure, either transcriptional repression or activation can occur [37]. H3K27me3 is associated with transcriptional silencing during mammalian embryogenesis [38]. H3K27me3 is normally catalyzed by the histone methyltransferase polycomb inhibitory complex 2 (PRC2) [39]. Some epigenetic factors are involved in the pathogenesis of AAA by regulating gene expression [40]. It is known that H3K27me3 is downregulated in Ang II-induced AAA tissues [37].

The article "EZH2 Regulates ANXA6 Expression via H3K27me3 and Is Involved in Angiotensin II-Induced Vascular Smooth Muscle Cell Senescence" was retracted in 2023. Reasons: signs of a paper mill; compromised peer review; unreliable results or conclusions.

EZH2 suppressed gene expression by adding a methyl group to histone H3 lysine 27, which promotes heterochromatin formation [41, 42]. Other research found that EZH2 is engaged in vascular diseases; for example, blocking EZH2 activity can effectively inhibit neointimal formation and vascular stenosis [43]. Li et al. [44] found that EZH2 promotes VSMC growth. Overexpression of EZH2 can increase the level of ANXA6 promoter H3K27me3, reduce the expression of ANXA6, inhibit the increase in ROS induced through Ang II and the senescence of VSMCs, and alleviate the pathogenesis of AAA.

In conclusion, we have shown that the expression of EZH2 was lower in rat AAA tissue and VSMCs could be induced by Ang II and the level of ANXA6 was increased in rat AAA tissue and VSMCs induced by Ang II. Overexpression of EZH2 reduced the level of ANXA6 by increasing the promoter H3K27me3 of ANXA6. Inhibiting Ang II-induced ROS increased VSMCs aging and alleviated the pathogenesis of AAA. It has been reported that the expression of EZH2 may be regulated by many factors, such as microRNAs and lncRNAs [45]. Therefore, we will examine the upstream mechanism of EZH2 in subsequent experiments. In addition, the regulatory mechanism of ANXA6 on ROS needs to be explored.

## 5. Conclusion

Our study shows that EZH2 regulates ANXA6 promoter H3K27me3 modification, inhibits ANXA6 expression, alleviates Ang II-induced VSMCs senescence, and inhibits AAA progression. This article will provide some theoretical significance for the treatment and diagnosis of AAA.

## Figures and Tables

**Figure 1:** ANXA6 expression is increased in AAA tissues. (a) Differential gene heat map between AAA patient abdominal aorta tissue and adjacent normal tissue. (b) Gene volcano map of the difference between AAA patient abdominal aortic tissue and adjacent normal tissue. (c) RT–qPCR for ANXA6 mRNA expression. (d, f) Assessment of ANXA6 expression in VSMC cells (d) and tissues (f) by Western blot. (e) Immunohistochemistry staining was used to assess ANXA6 expression. ^∗^*p* < 0.05, ^∗∗^*p* < 0.01.

The article "EZH2 Regulates ANXA6 Expression via H3K27me3 and Is Involved in Angiotensin II-Induced Vascular Smooth Muscle Cell Senescence" was retracted in 2023. Reasons: signs of a paper mill; compromised peer review; unreliable results or conclusions.

**Figure 2:** The influence of ANXA6 on Ang II-induced VSMCs senescence. (a) Western blotting for p16, p53, and p21 levels. (b) The mRNA level of IL-6 and IL-8 were assessed by RT–qPCR. (c) Flow cytometry for cell cycle. ^∗^*p* < 0.05, ^∗∗^*p* < 0.01. 2N represents G1 phase and 4N represents G2 phase in (c).

**Figure 3:** Knockdown of ANXA6 inhibits VSMC senescence by inhibiting the ROS production by Ang II-induced. (a) Assessing the effect of Ang II on ROS in VSMCs by Flow cytometry. (b) Western blot for p16, p53, and p21 levels. (c) The mRNA level of IL-6 and IL-8 mRNA were confirmed by RT–qPCR. (d) Flow cytometry for the cell cycle. ^∗^*p* < 0.05, ^∗∗^*p* < 0.01.

**Figure 4:** Knockdown of ANXA6 inhibits VSMCs senescence by inhibiting Ang II-induced ROS production in AAA rats. (a) Aneurysm representation of each group. (b) Aortic outer diameter of rats in each group. (c) Western blot for confirmed the level of p16, p53, and p21. (d) The mRNA level of IL-6 and IL-8 was confirmed by RT–qPCR. (e) Immunohistochemistry staining for ANXA6 expression. (f) Using *α*-SMA (green) and ANXA6 (red) double staining to confirm the level of ANXA6Z in VSMCs. (g) Using SA-*β*-gal staining was to assess the senescence of the aortic cells. (h) *α*-SMA (green) and p53 (red) double staining was used to assess the senescence of VSMCs in the aorta. (i) ROS levels in the aorta were assessed by DHE staining. (j) Hematoxylin and eosin staining to assess vascular lesions in the medial abdominal aorta. ^∗^*p* < 0.05, ^∗∗^*p* < 0.01.

**Figure 5:** The ANXA6 expression could be downregulated by EZH2 via H3K27me3. (a, b) In ANXA6 promoter, ChIP-qPCR was used to assess the expression of EZH2 and H3K27me3. (c) Western blot for confirmed by the influence of EZH2 on the expression of H3K27me3 and ANXA6. (d) RT-qPCR for confirmed the mRNA level of ANXA6. ^∗^*p* < 0.05, ^∗∗^*p* < 0.01.

**Figure 6:** EZH2 overexpression inhibits Ang II-induced ROS production by downregulating ANXA6 expression to inhibit VSMCs senescence. (a) ROS levels were assessed by flow cytometry. (b) The mRNA level of IL-6 and IL-8 were assessed by RT-qPCR. (c) Western blotting for p16, p53, and p21 expressions. (d) Flow cytometry for assessing the cell cycle. ^∗^*p* < 0.05, ^∗∗^*p* < 0.01.

**Figure 7:** EZH2 inhibits VSMC senescence in AAA rats by inhibiting ANXA6 expression. (a) Aneurysm representation of each group. (b) Aortic outer diameter of rats in each group. (c) Western blots for EZH2, ANXA6, p16, p53, and p21 expressions. (d) The mRNA level of IL-6 and IL-8 was confirmed by RT–qPCR. ANXA6 (e) and EZH2 (g) were assessed by immunohistochemistry staining. (e) *α*-SMA (green) and ANXA6 (red, f), EZH2 (red, h), or p53 (red, j). Using double staining to assess the level of AnxA6, EZH2, and p53 in VSMCs of arterial tssue. (i) Using SA-*β*-gal staining to detect the aging of aorticels. (k) ROS levels in the aorta were assessed by DHE staining. (l) Hematoxylin and eosin staining to assess vascular lesions in the medial abdominal aorta. ^∗^*p* < 0.05, ^∗∗^*p* < 0.01.

The article "EZH2 Regulates ANXA6 Expression via H3K27me3 and Is Involved in Angiotensin II-Induced Vascular Smooth Muscle Cell Senescence" was retracted in 2023. Reasons: signs of a paper mill; compromised peer review; unreliable results or conclusions.

## Data Availability

The data used to support the findings of this study are included within the article.

## Supplementary Materials

Supplementary Materials Figure S1: the representative ECG of the AAA patient. Figure S2: transfection efficiency test. The expression of ANXA6 was detected by Western blot after transfection of si-ANXA6 (A) and OE-ANXA6 (B). (C) The expression of EZH2 was detected by Western blot after transfection with OE-EZH2. ^ns^*p* > 0.05, ^∗∗^*p* < 0.01. Figure S3: effect of GSK126 on EZH2 expression. The expression of EZH2 was detected by Western blot. ^ns^*p* > 0.05.
